# Effect of Optimized Emergency Care on Treatment Rate and Prognosis of Elderly Patients with Acute Stroke in Emergency Department: A Systematic Review and Meta-Analysis

This article has been retracted.

**DOI:** 10.1155/2022/5841978

**Published:** 2022-07-26

**Authors:** Xia Liang, Yanhong Yu

**Affiliations:** ^1^Zhejiang Hospital Sandun Branch, The Emergency Department, Zhejiang, Hangzhou 310030, China; ^2^Zhejiang Hospital Sandun Branch, Geriatrics Department, Zhejiang, Hangzhou 310030, China

## Abstract

**Objective:**

This research was to detect the treatment rate and prognosis of elderly patients with acute stroke in emergency department by the optimization of emergency care applying meta-analysis.

**Methods:**

The online databases including PubMed, EMBASE, ScienceDirect, Cochrane Library, China knowledge Network Database (CNKI), China VIP Database, Wanfang Database, and China Biomedical Literature Database (CBM) were searched. The retrieval time limit was set from the establishment of the database to the present. The data were extracted independently by two investigators. The bias of per publication was assessed following Cochrane manual 5.1.0 standard. RevMan5.4 statistical software was used to analyze the collected data by meta.

**Results:**

The 8 randomized controlled trials included in this meta-analysis all reported patients' baseline status. The meta-analysis of the rescue time of the study group and the control group (CH2 = 1507.80, df = 4, *P* ≤ 0.001, and I2 = 100%) showed that the emergency nursing with optimized emergency procedures can shorten the rescue of elderly acute stroke patients in the emergency department time. There are 6 literatures reporting the case fatality rate (Chi^2^ = 1.12, df = 5, P = 0.95 > 0.05, and I2 = 0%), and the death rate of the study group was not higher than that of the control group (Z = 4.4 and *P* < 0.0001). The use of optimized first aid can reduce mortality in elderly patients with acute stroke. Six articles on disability rate reported the heterogeneity of disability rate (CH2 = 2.88, df = 5, *P* = 0.72 > 0.05, and I2 = 0%), indicating that the disability rate in the study group was lower than that in the control group (*Z* = 3.91 and *P* < 0.0001), indicating that emergency nursing by optimizing emergency procedures can reduce the disability rate of elderly stroke patients in emergency department.

**Conclusion:**

Optimizing the emergency care process can effectively improve the emergency rate and prognosis of elderly patients with acute stroke in emergency department; however, further research with higher methodological quality and longer intervention time are needed to verify later.

## 1. Introduction

With the rapid development of emergency medicine, prehospital first aid of acute stroke has become the focus. Rapid and standardized prehospital first aid can effectively reduce the rates of disability, mortality, and complications. Due to the constraints of prehospital first aid site conditions, most medical staff mainly make a preliminary differential diagnosis of patients based on patients' chief complaints, past medical history, and physical examination. After the initial diagnosis of stroke, the patients were given airway management immediately, and respiratory support was given to the patients through interventions such as oxygen therapy and balloon mask-assisted ventilation. In addition, for patients with acute ischemic stroke, vital signs should be monitored, and blood glucose monitoring should be carried out to help patients maintain supine position and tilt their head to one side, so as to prevent sputum or vomit from flowing back into the airway and causing ventricular breathing after prehospital first aid. The patients with acute ischemic stroke entered the hospital emergency department; in-hospital first aid became the key to treatment [1, 2]. The staff of the emergency department need to evaluate the patient's condition after the patient arrives and formulate a personalized treatment plan according to the actual situation of different patients, such as establishing venous access as needed, giving the patient oxygen or psychological counseling, and effective measures [3].

In the process of first aid for elderly patients with acute stroke, nurses participated in every link of first aid, such as emergency triage, rescue room, and transfer. However, the field of chest pain center certification experts did not fully realize the important position of nurses in the whole first aid process. However, the certification and evaluation standards for all aspects of the nursing process are still blank [4, 5]. At the same time, doctors still play a leading role in the optimization of first aid process for elderly patients with acute stroke in the emergency department; however, the nurses themselves do not fully realize the importance of improving the whole process. In addition, in the whole emergency process, most of the elderly patients with acute stroke in the emergency department are needed timely intervention measures by nurses in the process of first aid [6]. Medical staff ignore the humanistic needs of patients, thus further increasing the psychological burden of patients and reducing their compliance in the whole process of first aid. As a result, sometimes the first aid process is not smooth, and the treatment efficiency in the whole process is reduced [7, 8].

Professor Zhou Lanshu analyzed the significance and value of standardizing clinical nursing standards in her works and studied its necessity combined with the actual situation of clinical work [9]. Li Xiaofeng and Chen Min et al. [10] combined with previous research results improved the traditional rescue process, integrated nursing, and traditional medical first aid process and determined seven standardized nursing processes. The standardized nursing process can achieve early evaluation and early diagnosis, make the whole first aid process orderly, avoid repeated operations and unnecessary waiting time, and ensure the timeliness of rescue [11, 12]. In China, more and more attention has been paid to how to optimize the emergency nursing process for elderly patients with acute stroke in the emergency department. Wang Haiyan et al. [13] applied the quantitative standard matching model to the prehospital emergency nursing process and subdivided into five sub-processes. These five subprocesses make the nurses form a clear first-aid nursing idea and achieve a suitable and orderly seamless transformation. Previous analysis [14] through the establishment of chest pain optimization diagnosis and treatment team, the rescue time of elderly patients with acute stroke in emergency department decreased from 162.5 to 81.4, and the rate of reaching the standard of rescue time increased from 20% to 69.44% (all *P* < 0.01). At present, the literatures [15, 16] have proved that the optimized process of emergency nursing has a useful effect on the treatment rate and prognosis of elderly patients with acute stroke. However, the study has not been randomly assigned, and the sample size has been considered small and lack of credibility [17]. Therefore, this study quantitatively synthesized the published randomized controlled trials (RCT) by larger sample size.

## 2. Research Contents and Methods

### 2.1. Literature Retrieval Strategy

The retrieval strategy of the combination of subject words and free words was used to search PubMed, EMbase, The Cochrane Library, Web of Science, China Biomedical Literature Database, China knowledge Network, and Wanfang Database. The articles about emergency nursing for elderly patients with acute stroke were obtained from the establishment of the database to January 2022. The Chinese search words were set as follows: stroke, cerebral hemorrhage, cerebral ischemia, cerebrovascular accident, cerebral infarction, optimization of first aid flow, emergency nursing, and emergency nursing. The English search words were set to: stroke, cerebral hemorrhage, cerebral ischemia, cerebrovascular accident, cerebral infarction, optimization of first aid process, first aid nursing, and emergency nursing.

### 2.2. Inclusion and Exclusion Criteria

The inclusion criteria are as follows: (1) The type of study is RCT; (2) the subjects are senile acute stroke; and (3) the experimental patients accepted the first aid nursing which was optimized the first aid flow, and the control patients accepted the regular continuous nursing. The exclusion criteria are as follows: (1) non-Chinese and English literatures; (2) full text only describes random, but did not describe specific random methods; (3) unreported follow-up time; (4) intervention program combined with relevant theories; (5) literatures in which full or complete data could not be obtained.

### 2.3. Literature Screening and Data Extraction

Two researchers screened independently according to the standard retrieval strategy and inclusion and exclusion criteria. Different opinions were discussed with the third researcher and made the decision together. The researcher read through the entire text to extract author information, publication dates, basic information about the study population, specific intervention protocols, and outcomes.

### 2.4. Quality and Bias Risk Assessment of Included Literature

The bias risk assessment tool ROB2.0 for RCT recommended by Cochrane manual 5.1.0 was used to evaluate [18]. Two researchers independently evaluated the bias risk into the study and cross-checked the results.

### 2.5. Statistical Processing

The standardized mean difference (SMD) with Hedges' g was chosen as the measure of the effect. The effect size was calculated using a random-effects model with a restricted maximum-likelihood (REML) and considered a large, moderate, and small effect with respect to the SMD values of 0.8, 0.5, and 0.2, respectively. The heterogeneity among the studies included in a meta-analysis was assessed using Cochrane's Q, tau-squared, and I-squared (I2). Cochrane's Q test quantifies total variance and generates a *P* value that determines that the heterogeneity is present. Tau-squared indicates the true variance that is the between-study variance, while I2 represents the percentage of the total variance that is due to the true variance. The degree of heterogeneity is said to be low, moderate, and high, with I2 values of 25%, 50%, and 75%. RevMan 5.4 software was adopted for meta-analysis. HR and its 95% CI were employed as effect analysis statistics for OS and PFS, and risk ratio and 95% CI were employed as effect analysis statistics for binary variables. *P* and *I*^2^ values in heterogeneity test results were adopted to determine whether there was statistical heterogeneity among the results. *P* > 0.10 and *I*^2^ < 50% indicated that there was no statistical heterogeneity among the research results, and a fixed effect model was used for combined analysis. *P* ≤ 0.10 and *I*^2^ ≥ 50% indicated statistical heterogeneity among the research results, and a random effects model was adopted for combined analysis. The test level of meta-analysis was set as *α* = 0.05. Eggers' test was used to examine the funnel plot asymmetry. Whenever this test was significant with a *P* value of less than 0.1, we used the trim and fill method to correct the funnel plot and adjust the effect size for potential publication bias.

## 3. Results and Analysis

### 3.1. The Results of Literature Retrieval and the Basic Situation of Literature Inclusion

2941 articles were retrieved through computer database. 534 articles were obtained after eliminating repeated studies. 102 articles were obtained from preliminary reading of titles and abstracts. 43 articles were included after excluding irrelevant studies, reviews, case reports, and non-control literatures, and then 15 articles with incomplete data and no main outcome indicators were read carefully and finally included 8 RCT [19–26]. A total of 828 samples were analyzed by meta. The basic features included in the literature are shown in Table 1.

### 3.2. Evaluation of the Quality of the Methodology Included in the Literature

Only 3 RCT mentioned “random assignment” without any explanation, and the rest did not mention “random” information. Detailed intervention measures were given in all the 8 studies included. The number and reasons of blind method and loss of follow-up or withdrawal were not described in detail in 8 RCT articles. The evaluation of literature quality can be seen in Figures 1 and 2.

### 3.3. Meta-Analysis Result

#### 3.3.1. Rescue Time

Through the inclusion of 8 RCT studies, the rescue time between the study group and the control group was analyzed by meta. The heterogeneity test showed that Chi^2^ = 1507.80, df = 4, *P* ≤ 0.001, and *I*^2^ = 100%, indicating obvious heterogeneity. According to the results of this analysis, it can be considered that the emergency nursing care with optimized process can shorten the rescue time of acute elderly patients with acute stroke. The specific results are shown in Figure 3.

#### 3.3.2. Fatality Rate

Through the inclusion of 8 RCT studies, overall 6 articles reported the fatality rate. The heterogeneity test results were Chi^2^ = 1.12, df = 5, *P* = 0.95 > 0.05, and *I*^2^ = %, indicating no obvious heterogeneity. The fatality rate of the study group was lower than that of the control group (*Z* = 4.40 and *P* < 0.0001). It can be considered that the use of optimized emergency nursing can reduce the mortality of elderly patients with acute stroke. The specific results are shown in Figure 4.

#### 3.3.3. Disability Rate

Totally, 6 articles reported the disability rate and the disability rate was analyzed by meta. The heterogeneity test showed that Chi^2^ = 2.88, df = 5, *P* = 0.72 > 0.05, and *I*^2^ = 0%, suggesting no obvious heterogeneity. According to the results, the disability rate of the study group was lower than that of the control group (*Z* = 3.91 and *P* < 0.0001). It can be considered that the optimized process of emergency nursing can reduce the disability rate of elderly patients with acute stroke. The specific results are shown in Figure 5.

## 4. Discussion

Acute stroke is one of the most common diseases in the central nervous system, and it has a high morbidity and mortality rate, which seriously affects the prognosis of patients. The main manifestations of acute stroke are limb movement and speech dysfunction. In addition, it will also appear memory and cognitive function decline [27]. Ischemic stroke is the main type of acute stroke. It may bring serious and irreversible harm to the patients. The keys to treatment are to improve cerebral blood circulation [28]. It is considered that the time window for effective rescue of acute ischemic stroke is 4.5 to 6.0 hours. In order to win valuable rescue time, quick emergency nursing process is often adopted in clinic to improve the rescue effect of patients. Some studies have shown that the use of rapid nursing process in the rescue process of acute ischemic stroke can reduce the disability rate of patients and improve nursing satisfaction [29]. Therefore, in the process of rescue, it is necessary to improve the quality of nursing to appease patients.

In the past, the treatment of acute ischemic stroke mainly included blood pressure control, anticoagulant therapy, thrombolytic therapy, and vascular interventional therapy [30]. However, the majority of stroke patients presenting to the emergency department are in the acute phase. Therefore, it is more necessary to provide standardized nursing process for patients to avoid nurses' different practical experience and working habits. At present, the research on clinical nursing pathway of acute ischemic stroke in China is mainly focused on health education and psychological counseling, but the standardized and specific nursing process of integrated traditional Chinese and western medicine has not been formed in pre-hospital first aid and in-hospital emergency. At the same time, many human factors often appear in the process of prehospital first aid, resulting in the delay of the best time for treatment. The study of stroke pathway by Jiang Yunlan et al. confirmed that the implementation of clinical nursing pathway can effectively shorten the time of patients' visit [31]. An integrated Chinese and Western medicine pathway constructed for patients with hemorrhagic stroke, using a sequential treatment process to provide diagnostic, therapeutic and care measures by Wang Weiqiong [32]. It suggested the good effect has been achieved in the total effective rate of neurological function recovery and neurological function improvement after treatment in the path group. Xu Min [33] and others' researchers confirmed that the implementation of clinical pathway can significantly improve the neurological function of patients to improve the TCM syndrome differentiation and treatment ability of medical staff.

At present, meta-analysis confirmed that the effective diagnosis and treatment of acute ischemic stroke mainly include thrombolytic therapy, intravascular interventional therapy, antiplatelet therapy, anticoagulation therapy, and stroke unit [34]. Urokinase has become the main drug of thrombolytic therapy in China. At present, the Chinese guidelines for the diagnosis and treatment of Acute Ischemic Stroke (2014 Edition) believe that the time window for thrombolysis to rescue penumbra tissue is within 4.5 hours. At the same time, it is also pointed out in the guidelines that intravenous thrombolysis outside the time window is at risk of serious cerebral hemorrhage. However, the half-life of recombinant tissue-type plasminogen activator is only 3-5 minutes, which requires continuous intravenous drip [35]. Therefore, intravenous thrombolysis cannot be used as the only method for the treatment of acute ischemic stroke. Compared with intravenous thrombolytic therapy, endovascular interventional therapy is a therapeutic method to intervene the local thrombus directly, which can open the occluded vessels more quickly and effectively in theory. Its treatment mainly includes arterial thrombolysis, bridging therapy, mechanical thrombectomy, angioplasty, and stent thrombectomy, in which arterial thrombolysis and stent thrombectomy are also called intra-thrombotic therapy. Compared with intravenous thrombolysis, stent thrombectomy can significantly improve the recanalization rate. Studies have shown that the recanalization rate of stent thrombectomy can be as high as more than 90% [36]. It is confirmed that stent thrombectomy can not only improve the recanalization rate of occlusive vessels, but also effectively prolong the treatment time window. However, for patients with acute macrovascular occlusion within the thrombolysis time window, intravenous thrombolysis followed by intravascular interventional therapy is still the main means for the treatment of ischemic stroke. Whether endovascular intervention should be bypassed by intravenous thrombolysis is unclear. Some scholars believe that for patients with ischemic stroke caused by occlusion of large vessels in the anterior circulation, the therapeutic effect of combined intravenous thrombolysis and endovascular therapy within 4.5 hours is not better than direct endovascular intervention [37]. In recent years, a large number of studies on the application of recombinant pro urokinase in acute ischemic cerebral thromboembolism have confirmed that local intra-arterial perfusion of pro urokinase can achieve a higher vascular recanalization rate. However, the combined use of thrombolytic and anticoagulant drugs may lead to an increased risk of intracranial hemorrhage. In order to avoid the influence of thrombolytic and anticoagulant drugs on coagulation function, mechanical thrombectomy alone can rely on unique mechanical force to remove thrombus, thereby reducing the risk of intracranial hemorrhage.

The endovascular interventional therapy published in 2015 showed that compared with intravenous thrombolysis alone, endovascular interventional therapy based on intravenous thrombolysis can significantly improve the recanalization rate of occluded blood vessels [38, 39]. At the same time, the bleeding risk decreased after treatment, which further confirmed the efficacy and safety of endovascular interventional therapy in the treatment of acute ischemic stroke. Therefore, some scholars believe that endovascular interventional therapy is the second breakthrough in the field of ischemic stroke treatment following the application of recombinant tissue plasminogen activator to intravenous thrombolysis. In view of the high recurrence rate and high disability rate of patients with acute ischemic stroke, individualized antiplatelet and anticoagulation therapy should be given after admission. In addition to the guidance and intervention of stroke risk factors for different individuals, antiplatelet drugs are the main drugs for the prevention and treatment of local thrombosis in the stenotic site of ischemic stroke caused by atherosclerosis and stenosis of large arteries. According to the guidelines, patients with ischemic stroke who do not meet the indications for thrombolysis and have no contraindications should take aspirin as soon as possible after onset. A study of clopidogrel in the treatment of high-risk acute stroke group showed that [40] combined use of aspirin and clopidogrel for 3 weeks after transient ischemic cerebrovascular attack, compared with aspirin alone, can significantly reduce the 90-day deficit and the recurrence rate of hemorrhagic stroke. For cardiogenic stroke caused by atrial fibrillation, oral warfarin anticoagulation therapy can effectively reduce the risk of stroke. Although oral anticoagulants can effectively reduce the recurrence rate of ischemic stroke, statistics show that only about 45% of patients are treated with oral anticoagulants for a long time. According to the results of a study [41], about 38% of patients with ischemic stroke caused by atrial fibrillation are no longer treated with oral anticoagulants after discharge. The patients' survival rate with continuous oral anticoagulant therapy after 1 year was much higher than that of patients without anticoagulant therapy. In addition, recent studies also believe that improving targeted interventions in high-risk groups is of significant significance to reduce the recurrence of ischemic stroke. It has been proved that stroke unit (OR = 0.71) is the most effective measure in the diagnosis and treatment of ischemic stroke, which is better than thrombolytic therapy (OR =0.83) and antiplatelet therapy (OR = 0.99). It is a systematic and standardized management model for stroke treatment, which does not include new treatment methods [42].

The stroke unit mainly relies on close multidisciplinary links, with the participation of neurophysicians, professional nurses, physiotherapists, language rehabilitators, psychologists, social workers, and patients' families. Thus, we can formulate personalized diagnosis, treatment, and nursing programs for stroke patients in a planned and targeted manner, including timely and effective treatment measures, early rehabilitation training, prevention and treatment of complications, and other medical and nursing measures. However, due to the differences in the cognition of stroke and the constraints of medical level, medical system, and medical model, stroke units with practical clinical significance have not been formed in our country at present. For example, stroke patients in our country can generally get timely and effective drug treatment at the time of onset, but there is still a certain gap between the rehabilitation and prognosis programs in the later stage and those in developed countries [43].

The first aid nursing with optimized process can provide green first aid channel, abandon the traditional medical procedure of first registration before receiving, provide payment before treatment, save time for patients as far as possible, achieve seamless transmission of information, and be equipped with special personnel for guidance at the same time. It can also speed up patients' familiarity with the hospital structure and environment, which is helpful for patients' timely diagnosis and treatment [44]. At the same time, it can alleviate the negative emotions of patients and their families, avoid conflicts between panic and tension and medical staff, and save diagnosis and treatment time [45]. For patients with acute stroke, time is life; the earlier the rescue time, the earlier the recovery of cerebral blood supply, and the greater the probability of postoperative recovery. Some studies have shown that the disability and mortality of acute stroke patients with shorter rescue time are lower than those with longer rescue time [46]. In the rescue process of patients with acute stroke, doctors are often easy to ignore the various complications caused by rescue, so patients may have a variety of complications, affecting their follow-up treatment and rehabilitation process. Therefore, in the combined group, the nurses asked the patients about their conditions before the rescue and informed the doctors, which was helpful for the doctors to carry out predictive treatment during the rescue and reduce the occurrence of complications. Finally, 8 RCT articles were included in our investigation. All the 8 RCT literatures included in this meta-analysis reported the baseline status of patients, only 3 RCT mentioned “random assignment” without any explanation, and the rest did not mention “random” information. Detailed intervention measures were given in all the 8 studies included. The number and reasons of blind method and loss of follow-up or withdrawal were not described in detail in 8 RCT articles. Through the meta-analysis of the rescue time between the study group and the control group, heterogeneity test displayed Chi^2^ = 1507.80, df = 4, *P* ≤ 0.001, and *I*^2^ = 100%, showing an obvious heterogeneity among the collected researching data. This could be considered that emergency nursing with optimized emergency procedures could shorten the rescue time of elderly patients with acute stroke in the emergency department. A total of 6 articles reported the fatality rate, and heterogeneity test of fatality rate was Chi^2^ = 1.12, df = 5, *P* = 0.95 > 0.05,and *I*^2^ = 0%, indicating no significant heterogeneity. The death of the study group was not more common than the controls' death (*Z* = 4.40 and *P* < 0.0001), considering that the use of optimized emergency care could reduce the mortality of elderly patients with acute stroke. The 6 articles were reported about the disability rate; the heterogeneity test of the disability rate was Chi^2^ = 2.88, df = 5, *P* = 0.72 > 0.05, and I^2^ = 0%, suggesting no obvious heterogeneity. The disability rate of the study group was lower than that of the control group (*Z* = 3.91 and *P* < 0.0001), considering that the first aid nursing with optimized first aid flow can reduce the disability rate of elderly patients with acute stroke in emergency department. There are some limitations in this study. First of all, the sample size of the references included in this study is small, and they all belong to single-center research, and there is a certain deviation. In the future research, we will carry out a large sample of prospective studies and hopefully draw more valuable conclusions.

## 5. Conclusion

Optimizing the emergency care process can effectively improve the emergency rate and prognosis of elderly patients with acute stroke in emergency department; however, further research with higher methodological quality and longer intervention time are needed to verify later.

## Figures and Tables

**Figure 1:** Risk of bias assessment.

**Figure 2:** Risk of bias summary.

**Figure 3:** Forest plot of meta-analysis of rescue time between two groups.

**Figure 4:** Forest plot of meta-analysis of fatality rate between two groups.

**Figure 5:** Forest plot of meta-analysis of disability rate between two groups.

**Table 1:** Basic characteristics of literature.

Include the literature	Year of publication	N (C/T)	Intervention method		Random or not	Blind or not	Outcome index
			Control group	Research group			
Yuan Wenjing	2021	41/41	Routine nursing	Optimization of pre-hospital emergency nursing process	Not clear	No	①
Yang Wei	2017	25/25	Routine nursing	Emergency nursing fast track	No	No	①, ②, and ③
Song Yan	2017	27/27	Routine nursing	Emergency quick nursing process to implement nursing work	Yes	No	①,②, and ③
Wu Haixia	2016	108/117	Routine nursing	Emergency rapid nursing process	Not clear	No	①,②, and ③
Wang Juan	2022	43/44	Routine nursing	Optimize the process of emergency nursing	Yes	No	① and ②
Zhou Hongyan	2021	94/66	Routine nursing	Emergency quick nursing process	Not clear	No	① and ③
Ye Huishan	2021	40/40	Routine nursing	Emergency nursing green channel	No	No	①,② and ③
Cheng Yuhui	2021	45/45	Routine nursing	Emergency quick nursing process	Yes	No	①,②, and ③

Note: ① rescue time; ② fatality rate; ③ disability rate.

## Data Availability

The datasets used and analyzed during the current study are available from the corresponding author upon reasonable request.
